The article "Recurrence of a Rare Subtype of Guillain-Barré Syndrome Following a Second Dose of the Shingles Vaccine" was published in 2022. Journal: Cureus.

# Recurrence of a Rare Subtype of Guillain-Barré Syndrome Following a Second Dose of the Shingles Vaccine

**DOI:** 10.7759/cureus.30717

**Published:** 2022-10-26

**Authors:** Sikander Chohan, Ali Chohan

**Affiliations:** 1 Medical Education, Wayne State University School of Medicine, Detroit, USA; 2 Family Medicine, Western Michigan University Homer Stryker M.D. School of Medicine, Kalamazoo, USA

**Keywords:** gbs variant, neuromuscular disease, vzv, zoster vaccine, shingrix, guillain-barré syndrome

## Abstract

Guillain-Barré Syndrome (GBS) is an acute, immune-mediated polyneuropathy. The exact cause of GBS remains unknown, however, it commonly develops post-infection. Since the 1950s, various vaccines have been attributed to causing the syndrome, yet no definitive relationship has ever been determined. In 2021, the Food and Drug Administration (FDA) placed a black-box warning for Shingrix, a non-live recombinant vaccine against the varicella-zoster virus, regarding a possible risk of acquiring GBS post-vaccination in adults aged 65 and older. We report the recurrence of a rare subtype of GBS in a 61-year-old patient following the second dose of Shingrix. This case highlights the difficulty of diagnosing and treating recurrent GBS. It also raises awareness that Shingrix may be related to the development of GBS in younger patients. This case also emphasizes the importance of differentiating GBS from other polyneuropathies.

## Introduction

Guillain-Barré Syndrome (GBS) is an immune-mediated polyneuropathy. It is thought to be the most common form of acute, flaccid neuromuscular paralysis in the United States. Every year, there are one to two cases per 100,000 individuals, with the highest incidence in males [1]. The pathogenesis of GBS is the formation of immunoglobulin G (IgG) autoantibodies against gangliosides in myelinated axons of the peripheral nervous system. This demyelination, in turn, leads to the delayed transmission of impulses between neurons. 

About 70% of patients develop the syndrome after an infection [2]. Campylobacter jejuni (C. jejuni) is thought to be the most common preceding agent [3]. However, nonspecific viral pathogens that cause diarrheal illnesses may also be implicated. In turn, molecular mimicry, where antibodies against recently acquired infectious agents may react with gangliosides on neurons, may be involved in GBS [4].

GBS can present as differing variants. The most common variant in the United States, acute inflammatory demyelinating polyradiculopathy (AIDP), is characterized by lymphocytic infiltration of myelin [5]. Acute motor axonal neuropathy (AMAN) and acute motor and sensory axonal neuropathy (AMSAN) are rare variants that may occur due to molecular mimicry of axonal components. The former is characterized by motor impairment only, while the latter is characterized by motor and sensory weakness.

Most variants of GBS only affect the peripheral nervous system. Symptoms are characterized by progressive, bilateral weakness of the extremities. This leads to diminished deep tendon reflexes and ataxia. Sensory disturbances are nonspecific but include paresthesia, numbness, and impaired proprioception and vibration. There are four required criteria for the diagnosis of GBS: 1. progressive symmetric weakness of more than a single limb; 2. hyporeflexia or areflexia; 3. progression of symptoms in less than four weeks; 4. symmetric weakness [6-7].

An initial diagnosis of GBS is often made clinically. After admitting the patient, the next step is performing a lumbar puncture. Cerebrospinal fluid analysis commonly shows albuminocytological dissociation - an increase in protein count but normal lymphocyte count. The prevalence of this finding has an 80% sensitivity for the disorder [8]. A nerve conduction study can be performed. Electrodes are placed on the skin overlying a nerve and measure the speed of electrical impulses moving through neurons. Delayed F-waves, motor responses to nerve stimulations, and lower conduction velocities are characteristic of GBS. While this is the main diagnostic test done, electromyography (EMG) may also be performed. This measures the strength of impulses traveling to muscles. Diminished speed points to GBS and which specific variant the patient may have.

The most lethal complication of GBS is diaphragmatic weakness and subsequent respiratory failure. As such, frequent monitoring of vital capacities and inspiratory force is done [9]. If needed, the patient may be intubated and placed on mechanical ventilation. Plasma exchange (PLEX) or intravenous immunoglobulin G therapy (IVIG) is often done for patients experiencing debilitating weakness. PLEX directly removes antibodies and immune complexes in the plasma that may be causing GBS. IVIG’s role is less understood but is thought to impair antigen presentation, modulation of antibodies, and disruption of complement [5].

Shingles, known as Herpes Zoster, is an infection that occurs after varicella-zoster virus (VZV) reactivation. VZV is often acquired in childhood and can remain latent in the dorsal root ganglion. Immunosuppression (from other illnesses) or age-related immune system decline can lead to decreased protection against the virus, and subsequent reactivation [10]. The diagnosis of VZV is clinical, with the appearance of a painful, pustular rash in a dermatomal pattern.

In October 2017, the Federal Drug Administration (FDA) approved Shingrix, a non-live recombinant vaccine aimed to prevent shingles in adults 50 years and older. Administered in two doses, two to six months apart, the most common side effects are pain at the site of injection, muscle aches, and fever. In March 2021, the FDA placed a black box warning on Shingrix regarding the possible risk of acquiring GBS. A self-controlled case series found an increased risk of GBS during a 42-day period after vaccination with Shingrix [11]. The study also found an estimated three cases of GBS per million vaccinations administered in adults aged 65 and older [11].

This report illustrates the case of an elderly male who developed the rare acute motor sensory axonal neuropathy (AMSAN) variant of GBS. He recovered fully. Almost a year after his initial episode, the patient experienced a recurrence of the AMSAN variant of GBS following the administration of the Shingrix vaccine. The patient had no other illnesses or infectious exposures prior to his recurrence episode. Recurrent GBS is a rare phenomenon and difficult to diagnose. Limited literature exists on how the disorder presents and the risk factors associated with it. We hope to increase awareness of recurrent GBS and the possible link to vaccination with this case report.

## Case presentation

Initial episode

The patient was a 61-year-old with a past medical history of ​hypothyroidism, bipolar disorder, obstructive sleep apnea, hyperlipidemia, lumbar spine surgery, and right total knee replacement. Over the course of two weeks, the patient developed weakness in his body. He had recurrent, five-minute-long episodes of bilateral shaking of hands, which progressed to his entire body. His leg weakness and gait instability lead to three falls. The patient endorsed feeling particularly weak when standing and needing to support himself with a wall to remain upright. The patient denied experiencing vertigo, visual impairment, hearing loss, sensory impairment, headaches, or loss of consciousness. After visiting his psychiatrist, who noticed his weakness, he was encouraged to visit the emergency department (ED).

Upon arrival at the ED, the patient was admitted to neurology and underwent further workup. The patient denied recent illnesses, gastrointestinal issues, or travel outside his home state. Physical examination showed globally reduced pinprick sensation, reduced sensation to vibration bilaterally below the ankles, and impaired proprioception bilaterally below the ankles. The patient had absent deep tendon reflexes in the bilateral upper and lower extremities. Romberg sign was also present at the time of examination.

The patient had no abnormalities on an initial complete blood count, comprehensive metabolic panel, and urinalysis. All hormones and inflammatory mediators were within normal limits. ENA, ANA, anti-DSDNA, anti-GQ-1B, and anti-GQ-1C were negative. A paraneoplastic panel revealed no abnormalities. C. jejuni antibodies were negative. A lumbar puncture revealed albuminocytological dissociation-elevated protein with normal leukocyte count (Table 1). Nerve conduction and EMG were also done and pointed to a diagnosis of the AMSAN variant of GBS.

**Table 1:** Cerebrospinal Fluid Results From the Lumbar Puncture The patient had an elevated protein count. The leukocyte count, glucose, and lactic acid were within normal limits.

CSF Parameters	Patient’s Values	Reference
Protein	84	15-60 mg/dL
Leukocyte Count	4	0-5 mm^3^
Glucose	75	50-75 mg/dL
Lactic acid	17	10-25 mg/dL
Oligoclonal bands	Negative	Negative in GBS

The patient received five sessions of plasma exchange (PLEX) every other day over the course of one week. He received four total sessions. He gradually experienced an improvement in motor and sensory parameters. He was discharged after eight days with referrals to outpatient physical/occupational therapy and neurology.

Recurrence episode

Approximately 10 months later, the patient presented to his neurologist due to one week of difficulty walking. The patient endorsed feeling “wobbly” and unable to feel sensations in his fingers and toes. He also endorsed shortness of breath. Due to possible respiratory distress, his neurologist advised him to go to the emergency department. Upon arrival, the patient was again admitted. The patient denied recent illnesses, gastrointestinal issues, or travel outside his home state. The patient said he received a second dose of Shingrix two weeks before symptoms started. Since his symptoms presented nearly identically to the first episode, the patient was diagnosed with acute recurrent exacerbation of the AMSAN variant of GBS. He was monitored for respiratory distress with pulmonary function testing every eight hours.

Physical examination showed globally reduced pinprick sensation, reduced sensation to vibration bilaterally below the ankles, and impaired proprioception bilaterally below the ankles. The patient had absent deep tendon reflexes in the bilateral upper and lower extremities. Romberg's sign was unable to be assessed. The patient again received PLEX therapy daily for a total of four sessions. The patient experienced a complete improvement in motor strength. Sensation and reflexes continued to improve but had not yet returned to baseline. After five days of admission, the patient was discharged with recommendations to follow up with his neurologist.

## Discussion

Over time, the introduction of several new vaccines has subsequently led to an increase in reported GBS cases. However, to date, little concrete evidence exists proving vaccines can cause the syndrome. The 1976 influenza vaccine originated this association, with an estimated eight-fold increase in developing GBS [12]. Subsequent seasonal influenza vaccinations have not been associated with a risk of developing GBS [13]. After the introduction of the polysaccharide diphtheria toxoid conjugate vaccine (MCV4) in 2004, frequent reports of GBS occurring in children surfaced. Further studies have found no concrete association between the two [14]. The introduction of the measles/mumps/rubella, human papillomavirus, and rabies virus has also led to numerous case reports of post-vaccination GBS. No causal relationship has ever been found [14].

In addition to the primary trial that showed a modestly increased risk of developing GBS following Shingrix administration, there have been several case reports of this phenomenon. In 2019, one report described a 76-year-old female who developed the syndrome 10 days following her first dose of Shingrix [15]. Initial treatment with IVIG resulted in marked improvement; however, upon discharge, the patient re-experienced symptoms of GBS. Further treatment with PLEX resulted in a return to baseline. Another report from 2020 describes a 79-year-old male who developed GBS 10-days following Shingrix administration [16]. He was treated successfully with IVIG. Both reports are consistent with the primary trial, which found an increased risk in adults aged 65 and older who received the first dose [11].

Recurrence of GBS is defined as a second episode occurring at least two months after complete recovery from the first episode (or at least four months after partial recovery of the first episode) [17]. The recurrence rate is around 5% [18]. Patients with recurrent GBS are generally younger and usually present with the Miller-Fisher subtype [17]. Our patient had the AMSAN variant in both episodes. Treatment of recurrent GBS is similar to initial treatment, focusing on protecting airways and administrating PLEX or IVIG. Treatment of GBS following vaccination remains identical as well.

Limited research exists on how similar or severe recurrent GBS is to the initial episode. Studies from the 1990s generally found that recurrent episodes can be severe with possible respiratory impairment [18]. However, a study from 2020 found most patients to have a mild second episode [17]. Our patient had similar symptoms in each episode. His second episode presented with some respiratory distress in addition to previous symptoms similar to the previous episode.

This case also highlights the importance of distinguishing recurrent GBS from GBS with treatment-related fluctuation (GBS-TRF) and chronic inflammatory demyelinating polyneuropathy (CIDP), as each is treated differently. GBS-TRF, which can occur in up to 15% of patients, there is post-treatment improvement in symptoms and then redevelopment of symptoms within two months [17]. It may occur due to lasting immune system activation and too early initiation of therapy [19]. Patients with these cases are usually given specific, tailor-made treatments. Similar to GBS, CIDP is a demyelinating autoimmune disease where symptoms slowly worsen and persist longer than eight weeks [19]. It is treated with steroids.

Future studies should focus on determining whether there are links between the triggers for the initial and recurrent GBS episodes. This relationship may provide valuable insight into what causes the syndrome to develop. Insight into the clinical presentation of recurrent GBS must also be further studied. Determining how similar it presents to the initial episode, which treatments are appropriate, and if there are any potential triggers will provide insight into how to treat the syndrome. Determining whether Shingrix is associated with GBS in younger patients is of utmost importance. Our patient was younger than the demographic the FDA released a black box warning for. As we learn more about GBS and its causes, we will better understand any link to vaccines and can provide adequate care to patients suffering from it.

## Conclusions

The limitations of this report include potential exposures to risk factors of GBS that the patient may have been exposed to in the time period between his first and second episodes. Additionally, recurrent GBS is still poorly understood and its relationship to Shingrix is actively being researched. To our knowledge, this is the first case of GBS recurrence following vaccination with Shingrix. Relatively little data exist regarding GBS recurrence risk after vaccination. Officially, the CDC recommends precautions for patients with a history of GBS receiving certain vaccinations. In general, providers are recommended to educate the patient on the efficacy and benefit of vaccines and monitor for any potential GBS-like symptoms following vaccination. Clinicians should be specifically cautious for patients of any age, with a past history of GBS, who are receiving the Shingrix vaccine. In terms of treatment, clinicians should also be aware that the regimen remains identical to the initial episode. When presented with a recurrence of GBS, clinicians must also definitively rule out GBS-TRF or CIDP before administering treatment.
